The article "The Expression of hnRNP A2/B1 in Benign and Malignant Lung Lesions and Its Early Diagnosis Value in NSCLC" was retracted in 2023. Reasons: unreliable results or conclusions; lack of ethics approval or compliance; concerns about the data; concerns about the peer review.

# The Expression of hnRNP A2/B1 in Benign and Malignant Lung Lesions and Its Early Diagnosis Value in NSCLC

**DOI:** 10.1155/2022/5687245

**Published:** 2022-10-05

**Authors:** Wenchao Gu, Xiwen Gao, Linxun Wang, Guoping Deng, Jiaru Huang, Junxia Yang, Yuan Liu, Qun Liu, Hongyang Sang

**Affiliations:** ^1^Department of Respiratory Medicine, Shanghai Pudong New Area People's Hospital, Shanghai 201200, China; ^2^Department of Pulmonary and Critical Care Medicine, Minhang Hospital, Fudan University, Shanghai 266119, China; ^3^Neurology Department, Lianshui County People's Hospital, Lianshui 223400, China; ^4^Department of Cardiothoracic Surgery, Shanghai Jiaotong University Affiliated Sixth People's Hospital, Shanghai 201306, China

## Abstract

Lung cancer in its occurrence and development of different stages exist different biological behavior changes. This paper studies the expression of heterogeneous nuclear ribonucleoprotein (hnRNP) A2/B1 in benign and malignant lung lesions and its early diagnosis value of nonsmall-cell lung cancer (NSCLC), aiming to provide reference for the early diagnosis and therapy of NSCLC. Some lung surgery specimens are selected from January 2021 to March 2022. All cases received no radiotherapy and chemotherapy before surgery, including 90 sufferers with benign lung lesions as the contrast set. hnRNP A2/B1 expressions are measured for comparison. The experimental results show that for lung cancer sufferers, the positive expression of hnRNP A2/B1 in their malignant lesion tissue is notoriously higher than that in their benign lesion tissue, and hnRNP A2/B1 is differently expressed in different differentiation and in different stages.

## 1. Introduction

Like other malignant tumors, lung cancer has different biological and behavioral changes in different stages of its development, including precancerous lesions and early carcinogenesis, whether in the clinical manifestations [1]. The cell biological behavior is obviously different from the late tumor stage. Therefore, it is important to deeply understand the biological behavior characteristics, regularity, and molecular tumor markers to enhance the early diagnosis rate of lung cancer and enhance the therapy effect of lung cancer [2]. Lung cancer is one of the most common malignancies, and its incidence and mortality remain on the rise. However, as one of the most insidious ailments, the early diagnosis of lung cancer is difficult, and the traditional sputum cytology affects its clinical application due to its low detection rate [3, 4].

Recent studies have shown that heterogeneous nuclear ribonucleoprotein (hnRNP) A2/B1 is overexpressed in early lung cancer and precancerous lesions and can be detected by sputum examination, and its relationship with nonsmall-cell lung cancer (NSCLC) has gradually attracted clinical attention [5, 6]. This paper studies the expression of hnRNP A2/B1 in benign and malignant lung lesions and its early diagnosis value of NSCLC, aiming to provide reference for the early diagnosis and therapy of NSCLC.

The article "The Expression of hnRNP A2/B1 in Benign and Malignant Lung Lesions and Its Early Diagnosis Value in NSCLC" was retracted in 2023. Reasons: unreliable results or conclusions; lack of ethics approval or compliance; concerns about the data; concerns about the peer review.

The rest of this paper is organized as follows: Section 2 discusses related work, followed by cases information, and examination methods designed in Section 3.  Section 4 shows the experimental results and analysis, and Section 5 is the conclusion, which briefly summarizes all of the standpoints of the paper.

## 2. Related Work

Many studies have shown that lung cancer development is a multistage and multistep occurrence process. Prior to the morphological alterations, there have been many changes in molecular biology, such as the activation of protooncogenes and the inactivation of tumor suppressor genes [7]. Therefore, understanding the initial molecular events leading to lung cancer development may enhance our ability to predict the risk of lung cancer occurrence and provide new strategies for its early diagnosis and therapy [8]. In recent years, studies have found that hnRNP A2/B1 is overexpressed in early lung cancer and precancerous lesions, and it can be detected by sputum examination, which has a higher sensitivity than previous cytomorphological examination, and many studies support the overrepresentation of hnRNP A2/B1 as an early event of lung cancer formation [9].

The results of a series of studies suggest the selective expression of the hnRNPs family in lung cancer, especially the high expression of hnRNP A2/B1 in lung cancer. In this examination, the expression of the lung cancer cell lines was examined by applying immunohistochemistry, western blot, and PCR. The positive expression of hnRNP A2/B1 in malignant lesion tissues was found in 76.67% of lung cancer, and it was notoriously higher than 22.22% (*P* < 0.05). As the expression standard of hnRNP A2/B1 is closely associated with cell proliferation, and relative to permanently surviving normal cell lines, with the same hnRNP A2/B1 expression standards as in the tumor cell lines, so it is very difficult to find suitable normal cell lines in a short clinical time [10]. Therefore, contrast to the established lung cancer cell lines or primary cultures, lung cancer is best studied by biopsy tissue specimens. Related examination data suggest that on the protein standard and gene standard, hnRNP A2/B1 expression in lung cancer, can be used as an important feature of new cells to morphological differentiation, has an important significance for the early diagnosis of lung cancer [11]. HnRNP A2/B1 is expressed at very low or even no expression standards in normal bronchial epithelial cells, but is elevated in the central airway and metaplastic epithelial tissues of chronic smokers and notoriously subjoined in lung cancer tissues. The examination believe that this phenomenon may be that the expression standard of hnRNP A2/B1 during cell proliferation is regulated by differentiation in different cell proliferation stages, causing lung cancer due to regulatory disorders [12, 13]. The present examination found that with the increase of the stage, its positive expression rate was notoriously subjoined, and there is an extensive disparity. HnRNP A2/B1 positive expression was notoriously higher in the poorly differentiated set than in the moderately differentiated and highly differentiated sets. The disparity was statistically extensive (*P* < 0.05). As it is reported in the literature, hnRNP A2/B1 can be widely expressed in malignant lesions and proliferating cells in the early or premalignant stages of lung cancer. hnRNP A2/B1-positive cells with microsatellite changes and heterozygosity deficiency had a three-times higher frequency than those of cells with negative cells for the hnRNP A2/B1 expression [14]. Sputum examination of sufferers with suspected lung cancer found that 65% of those with the high hnRNP A2/B1 expression developed a lung cancer knife within 1 year. Therefore, it shows that hnRNP A2/B1 molecule may be an early event of lung cancer, and a further examination of the role of hnRNPA2B1 in the development of lung cancer can help to find early lung cancer sufferers, effectively enhance the early diagnosis rate of lung cancer, increase the chance of surgery, and reduce the case of fatality rate [15]. However, the participating sufferers were not followed up in this examination, so their long-term situation cannot be determined, and further examination is needed in future studies.

The article "The Expression of hnRNP A2/B1 in Benign and Malignant Lung Lesions and Its Early Diagnosis Value in NSCLC" was retracted in 2023. Reasons: unreliable results or conclusions; lack of ethics approval or compliance; concerns about the data; concerns about the peer review.

In addition, through the decomposition of the value of NSCLC assessed by hnRNP A2/B1, we found that the area of the receiver operating characteristic (ROC) curve was 0, with a high specificity of 82.20% and a sensitivity of 87.50%. The main reason was that hnRNP A2/B1 is an important RNA-connecting egg. White, is the basic core component of the hnRNP in the nucleus. Moreover, hnRNP protein and RNA bind to a certain degree of sequence specificity, shuttling between the nucleus and cytosol, participating in mRNA transport and posttranscriptional regulation, and has the functions of preventing RNA degradation [16]. Furthermore, hnRNP A2/B1 binds to telomeric single strands in a random manner, protecting it from nuclease breakdown and activating telomerase, while overexpression in cancer cells and proliferating cells, may be a cause of cell carcinogenesis. hnRNP A2/B1 is overexpressed in critical stages of normal lung development, with expression standards similar to lung cancer and precancerous lesions, and its expression in the mature lung tissue is suppressed and seen in lung cancer similar to embryonic lung growth, which is almost consistent at protein and signaling molecular standards, suggesting that hnRNP A2/B1 may be a possible oncodevelopment protein[17].

## 3. Cases Information and Examination Methods

### 3.1. Cases Information

Lung surgery specimens from some NSCLC patients in our hospital from January 2021 to March 2022 are selected. All cases did not receive radiotherapy or chemotherapy before surgery. There are 90 cases in all: 70 males and 20 females, aged 28 to 76 years, mean age(58.73 ± 10.59) years; 28 cases of squamous cell carcinoma, 42 cases of adenocarcinoma, and 42 cases of adenosquamous cell carcinoma, 20 cases of cancer; 18 cases of poorly differentiated carcinoma, 22 cases of moderately differentiated carcinoma, and 50 cases of well-differentiated carcinoma. P-TNM staging (international UICC1997 staging standard) are as follows: 7 cases of stage IA, 21 cases of stage IB, 13 cases of stage IIA, 19 cases of stage IIIB, 22 cases of stage IIIA, and 8 cases of stage IV. A total of 90 patients with benign lung lesions who received physical examination in our hospital during the same period are selected as the control group. Lung cancer tissues are obtained from lung tumors, and adjacent lung tissues are obtained from lung tissues with normal pathological examination more than 5 cm away from the tumor. All patients included in the study signed the informed consent form. The treatment methods and detection methods used in this study are all known safe methods in the clinic. The general information and clinical data collected in this study are only used for research analysis, not for other uses. If you have any discomfort during the treatment, please inform your doctor in charge in time to decide the next treatment plan. During the entire treatment period, please inform the doctor of the changes in your condition in time. Other medicines and other treatments, if used, please inform your physician.

### 3.2. Examination Methods

#### 3.2.1. Main Reagents

The sheep antihuman hnRNP A2/B1(G 16)\sc-10036 polyclonal antibody is purchased from Santa Cruz Biotechnology. The biotinylated rabbit antisheep antibody (c anti) and streptomycin-biotin-one-peroxide complex are purchased from Beijing Zhongshan Biology (SP-9003 HistostainTM-Plus kits) [18].

The article "The Expression of hnRNP A2/B1 in Benign and Malignant Lung Lesions and Its Early Diagnosis Value in NSCLC" was retracted in 2023. Reasons: unreliable results or conclusions; lack of ethics approval or compliance; concerns about the data; concerns about the peer review.

#### 3.2.2. Methods

Immunohistochemical staining is performed by the streptomycin probiotic monophenol oxidase method (S-P method). Paraffin-embedded tissue to be measured is cut into 5 pm thick sections [19, 20]. Xylene and gradient alcohol are dewaxed to water, 3% hydrogen peroxide (H2O2) blocking the endogenous peroxidase, high-pressure repair of the antigen, and 3% normal rabbit serum is incubated for 30 min to seal nonspecific antigens; incubation with the anti-hnRNP A2/B1 mAb (1 : 100) at 4°C overnight. After shock washing with 0.01 mol/L of P B S buffer, we should add the biotinylated secondary antibody working solution (rabbit antisheep), 37°C for 40 min; PBS shock washing, drop streptomycin-biopro monoperoxide complex working solution, 37°C for 30 min; PBS shock washing, DAB coloration, hematoxylin redye; 2% Z alcohol hydrochloride, 1/500 water reverse blue, dehydration transparent sealing. The negative contrast uses PBS instead of the primary antibody, other steps are the same.

By the ELISA method, hnRNP A2/B1 (G 16) kit (Beijing Zhongshan Biology), the detailed steps are as follows: add a blank hole (without sample and labeling reagent and the same steps) for the test sample hole; add 40 l of sample dilution to the test sample hole on the coated plate and then 10 l of the sample for the test (the final dilution of the sample is 5 times); add the sample to the bottom of the microplate hole, try not to touch the hole wall, gently shake and mix well; add enzyme, 100 l of HRP-mapping reagent is added to each well, except for the blank holes; heating and incubation: seal the plate with sealing plate film after 37°C heating and incubation for 60 minutes; distribution liquid: dilute the 20 times concentrated washing liquid with distilled water 20 times for backup; washing: carefully remove the sealing plate film, leave the liquid, spin dry, fill each well with the wash solution, leave for 30 seconds, this is repeated 5 times, and beat the dry; color development: add A 50 *μ*l to each well, add back to the color developer B 50 *μ*l gently, at 37°C for 15 min, then data decomposition software is used for data decomposition.

#### 3.2.3. Judgment of Immunohistochemical Results

In a double-blind manner, 5 to 10 visual fields and 100 to 200 cells are counted under a high magnification lens (400) per slice, for a total of 1,000 cells. The bronchial epithelium with low cell count have 200 cells. By staining intensity, 0 is one, 1+, 2++, and 3+++. Then the proportion of stained positive cells is calculated respectively: 0 is divided into no positive cells, 1 into positive cells <10%, 2 into positive cells 10%∼50%, and 3 into positive cells >50%. Staining index (SI) = the sum of the two, SI >2 is regarded as positive immunostaining, 0∼2 into one, 3 to 4 as+, 4-5 as++, and 6 as+++; 85% of cells are cytoplasmic and cytokaryotype.

The article "The Expression of hnRNP A2/B1 in Benign and Malignant Lung Lesions and Its Early Diagnosis Value in NSCLC" was retracted in 2023. Reasons: unreliable results or conclusions; lack of ethics approval or compliance; concerns about the data; concerns about the peer review.

#### 3.2.4. Observation Indicators

There are five observation indicators which are as follows:

1. Observe the hnRNP A2/B1 immunohistochemical maps in different tissues;
2. Disparity in the hnRNP A2/B1 positive expression in benign and malignant lesions;
3. hnRNP A2/B1 positivity is expressed in different stages;
4. hnRNP A2/B1 positivity is expressed in different differentiation;
5. The diagnostic value of hnRNP A2/B1 in NSCC lung cancer.

### 3.3. Statistical Methods

First, the excel form is established, organize the data required for the examination in sets, and open SPSS 26.0 to analyze the data separately. Measurement data representation and test methods are *n* (%) and 2, respectively, analyze correlation by Pearson and use the ROC curve when *P* < 0.05.

## 4. Experimental Results

### 4.1. Organization Distribution

Figure 1 shows the distribution of different tissues and hnRNP A2/B1 distribution. It can be seen from Figure 1 that hnRNP A2/B1 is correspondingly expressed in both the nucleus and the cytoplasm, mainly expressed in the nucleus, less expressed in the cytoplasm, and almost not expressed in the cell membrane. The high expression rate of squamous carcinoma, adenocarcinoma can also appear high expression, adjacent bronchial mucosa mucus glands also have corresponding expression, and benign mass have less expression or basically no expression. The statistical results show that hnRNP A2/BI is highly expressed in lung cancer tissues and also in the para bronchial mucosa, suggesting that hnRNP A2/BI may occur at the initiation stage of lung cancer and may be related to the occurrence of lung cancer.

### 4.2. Contrast of hnRNP A2/B1 Expression in Benign and Malignant Lung Cancer Tissues

Table 1 shows the contrast of the hnRNP A2/B1 expression in benign and malignant lesions of lung cancer.  Figure 2 shows the comparison of the hnRNP A2/B1 expression in benign and malignant lung cancer tissues. It can be observed from Table 1 and Figure 2 that the positive expression of hnRNP A2/B1 in malignant lesions of lung cancer is 76.67%, which is notoriously higher than in 22.22% (*P* < 0.05).

### 4.3. The hnRNP A2/B1 Expression in Different Stages of Lung Cancer

Table 2 shows the disparity in the hnRNP A2/B1 expression in different stages of lung cancer. It can be seen from Table 1 that the expression of hnRNP A2/B1 varied notoriously in different lung cancer sufferers at different stages, mainly showing the increase of the positive expression rate with extensive disparities (*P* < 0.05).

The article "The Expression of hnRNP A2/B1 in Benign and Malignant Lung Lesions and Its Early Diagnosis Value in NSCLC" was retracted in 2023. Reasons: unreliable results or conclusions; lack of ethics approval or compliance; concerns about the data; concerns about the peer review.

### 4.4. The hnRNP A2/B1 Expression in Different Differentiation of Lung Cancer

Table 3 shows the differential hnRNP A2/B1 expression in different differentiation of lung cancer. It can be seen from Table 3 that the positive expression of hnRNP A2/B1 is notoriously different in the different differentiation of lung cancer, mainly manifested by the notoriously higher positive expression of hnRNP A2/B1 in the less differentiated set than in the middle and highly differentiated sets, which is statistically extensive (*P* < 0.05).

### 4.5. Decomposition of hnRNP A2/B1 in Non-SCLC

Table 4 shows the diagnosis value of hnRNP A2/B1 for NSCLC.  Figure 3 shows the ROC curve of the early diagnostic value of hnRNP A2/B1 used in non-SCLC. Through the above experimental results, it can be observed that the area below the ROC curve for hnRNP A2/B1 assessment is 0, with a high specificity of 82.20% and a sensitivity of 87.50%.

## 5. Conclusion

The expression of heterogeneous nuclear ribonucleoprotein (hnRNP) A2/B1 in benign and malignant lung lesions and its early diagnosis value of NSCLC is studied. For lung cancer sufferers, the positive expression of hnRNP A2/B1 in their malignant lesion tissue is notoriously higher than that in their benign lesion tissue, and hnRNP A2/B1 is differently expressed in different differentiation and in different stages, which has a high diagnostic value for nonsmall-cell lung cancer.

## Figures and Tables

**Figure 1:** Distribution of different tissues and hnRNP A2/B1: (a) moderately differentiated adenocarcinoma; (b) moderately differentiated squamous carcinoma; (c) adjacent tissue; and (d) inflammatory pseudomonatissue.

**Figure 2:** Comparison of the hnRNP A2/B1 expression in benign and malignant lung cancer tissues.

**Figure 3:** The ROC curve of the early diagnostic value of hnRNP A2/B1 used in non-SCLC.

**Table 1:** Contrast of the hnRNP A2/B1 expression in benign and malignant lesions of lung cancer.

Sets	hnRNP A2/B1				Positive
	−	+	++	+++	
The tissue of malignant lesions (*n* = 90)	21	23	27	19	69 (76.67)
The benign lesion tissue (*n* = 90)	70	15	5	0	20 (22.22)
*χ* ^2^					12.633
*P .*					<0.001

**Table 2:** disparity in the hnRNP A2/B1 expression in different stages of lung cancer.

Sets	hnRNP A2/B1				Positive
	−	+	++	+++	
Phase IA (*n* = 7)	4	2	1	0	3 (42.86)
Phase IB (*n* = 21)	7	7	5	2	14 (66.66)
Phase A (*n* = 13)	4	6	1	2	9 (69.23)
Phase B (*n* = 19)	4	2	9	4	15 (78.95)
Phase A (*n* = 22)	2	4	12	4	20 (90.91)
Period (*n* = 8)	0	0	1	7	8 (100.00)
*χ* ^2^					16.271
*P*					<0.001

**Table 3:** differential hnRNP A2/B1 expression in different differentiation of lung cancer.

Sets	hnRNP A2/B1				Positive
	−	+	++	+++	
Highly differentiated carcinoma (*n* = 50)	15	15	20	0	30 (60.00)
Median-differentiated carcinoma (*n* = 22)	5	5	7	5	17 (77.27)
Low-differentiated carcinoma (*n* = 18)	1	3	0	14	17 (94.44)
*χ* ^2^					14.653
*P*					<0.001

The article "The Expression of hnRNP A2/B1 in Benign and Malignant Lung Lesions and Its Early Diagnosis Value in NSCLC" was retracted in 2023. Reasons: unreliable results or conclusions; lack of ethics approval or compliance; concerns about the data; concerns about the peer review.

**Table 4:** diagnosis value of hnRNP A2/B1 for NSCLC.

Metrics	Accuracy	Sensitivity	Specificity	Cutoff values (%)	AUC
Joint detection	87.00	87.50	82.20	93.25	0.827 (0.729∼0.852)

## Data Availability

The simulation experiment data used to support the findings of this study are available from the corresponding author upon request.
